# A Tropical Cyclone Center Location Method Based on Satellite Image

**DOI:** 10.1155/2022/3747619

**Published:** 2022-03-08

**Authors:** Qingxiang You, Zhenqing Li, Cheng Qian, Tian Wang

**Affiliations:** ^1^Department of Computer and Information Engineering, Changzhou Institute of Technology, Changzhou, China; ^2^University of Shanghai for Science and Technology, Shanghai, China

## Abstract

Accurately detecting and locating the center of the tropical cyclone is critical for the trajectory forecasting. This study proposed an automatic method for centers' location of the tropical cyclones based on the visible or the infrared satellite images. The morphological structure of the tropical cyclone is modeled using the circular pattern. The tropical cyclone center is located based on regional pixels instead of skeleton points. All pixels in a segmented cloud cluster vote for a 2-dimensional accumulator. The center of the cloud cluster is computed by the mean voting distances, which are calculated by fitting quadratic functions in every column of the two-dimensional (2D) accumulator. Then, a linear function is fitted according to the functional relationship between the mean voting distance and voting angle. The fitted coefficients of the linear function are the center coordinates of the tropical cyclone. The proposed method for centers location of the tropical cyclones is tested using visible and infrared satellite images. The results of center location are compared with the best track provided in JMA datasets.

## 1. Introduction

The tropical cyclone is a kind of atmospheric circulation systems, which may cause disasters and lead to economic loss in coastal areas. The trajectory forecast [1, 2] of tropical cyclones is very significant in order to avoid the destruction by tropical cyclones. Meteorological satellites offer a reliable solution to observe tropical cyclones [3, 4]. The trajectory of a tropical cyclone can be analyzed and estimated based on satellite images [5]. The first comprehensive technique for analyzing tropical cyclones using satellite images was Dvorak techniques [6].

The center location for a tropical cyclone is important for the trajectory forecast of the tropical cyclone [7–9]. The center position of the tropical cyclone is estimated by finding the spiral origin [10] or by fitting the elliptic center [11]. Huadong et al. [12] and Ryglicki and Hart [13] investigated various methods of tropical cyclone center location and classified methods into two categories: morphological pattern analysis method and wind field analysis method.

The first kind of method is based on pattern analysis of morphological characteristics of the tropical cyclone [14, 15]. By using image processing techniques [16], the spiral center of the cyclone is determined by finding the origin of a logarithmic helix [17] or by locating the point where the gradient vectors of brightness temperature are converging [18]. In order to detect the tropical cyclone center, the density matrix [19] and the deviation angle variance [20] are exploited. The located center is accurate, but it does not work well when the morphological structure of the tropical cyclone is not apparent.

The second kind of method is based on the wind field analysis [21, 22]. The center of tropical cyclone is determined by finding the minimum value of wind speed or the maximum value of cyclone vortices [23]. In order to locate the center position of the tropical cyclone, a mathematical morphology method [24] or saliency detection method [25] are utilized. It can deal with the center location of weak circulation, but the wind field inversion is affected.

The current methods for center location of the tropical cyclone require applying an edge detector to extract skeleton points in satellite cloud images. However, the extracted skeleton is usually inaccurate due to noise and disturbance. The tropical cyclones are often segmented from the images before the circle detection, so the shape of the tropical cyclone relies on the segmentation result. When the noise is incorporated into the segmentation result, the shape of the tropical cyclone is distorted. The circular skeleton is not enough definite for the successive circle detection. It will lead to the failure in the circle detection. In order to overcome the problem of edge extraction, the tropical cyclone center is analyzed and located based on regional pixels instead of skeleton points. The methods based on Hough transform can be used to detect circles [26, 27]. The voting of parameters determines the locations and the sizes of the circles. Using a modified Hough transform [28], the center position of the tropical cyclone is determined by fitting a linear function according to the functional relationship of the mean voting distance, which is calculated in each column of the accumulator by fitting a quadratic function.

## 2. Methods

The satellite cloud image is segmented; firstly, the segmented cloud cluster with the most pixels is selected. After regional pixels' vote, the center of a cloud cluster is determined by function fitting techniques. The proposed algorithm is made up of four steps: image binarization, Hough vote, searching voting distances, and solving the center coordinates. The flowchart of the proposed algorithm is shown in Figure 1.

### 2.1. Satellite Cloud Image Segmentation

The image is segmented using seed expanding and the threshold constraint [29–31]. Two thresholds are defined. The first threshold T1 is defined as the quantity of pixels whose intensity greater than T1 is less than 300. The second threshold T2 is defined as the quantity of pixels whose intensity greater than T2 is less than 30000. A pixel, whose intensity is greater than T1, can be selected as a seed. If the intensity of its neighboring pixel is greater than T2, the region is expanded [32].

The region with the most pixels is considered as a candidate of the tropical cyclone. An example of cloud image segmentation is shown in Figure 2. Although the shape of a segmented cloud cluster is irregular, it is modeled using a near-circular pattern. The circle center is considered as the center of a cloud cluster corresponding to a tropical cyclone.

### 2.2. Regional Pixels' Voting

In order to extract the center of the near-circular cloud cluster, a modified Hough transform is used. Instead of skeleton points, the regional pixels vote for a 2-dimensional accumulator. The voting formula is

(1) $$\begin{array}{c} \rho =x\cdot \cos\;\theta +y\cdot \sin\;\theta ,\;\theta \in \left[\begin{array}{cc} 0 & \pi \end{array}\right), \end{array}$$

where *θ* is the Hough voting angle and *ρ* is the computed voting distance. For a voting angle *θ*_*i*_, the validated voting distance *ρ* is limited. It is shown in Figure 3. *ρ*_*m*_ is the mean voting distance with respect to each voting angle *θ*. It is also the regional center voting for the 2D accumulator. The voting value *H*(*θ*,*ρ*) increases from 0 to the maximum and then decreases to 0. Let *ρ*_*m*_(*θ*) be the mean voting distance corresponding to the voting angle *θ*.

After all regional pixels have voted for the 2D accumulator, a quadratic function is fitted using the voting information in each column of the 2D accumulator.

### 2.3. Quadratic Functions' Fitting

The voting value *H*(*θ*,*ρ*) corresponding to distance *ρ*_*j*_ and angle *θ*_*i*_ is illustrated in Figure 4. The voting value is

(2) $$\begin{array}{c} H\left(\rho ,\theta \right)=2\cdot \sqrt{r^{2}-{\left(\rho -\rho_{m}\right)}^{2}}. \end{array}$$

Thus, the functional relationship of the voting value *H*^2^(*θ*,*ρ*) with respect to the voting distance *ρ* is a quadratic polynomial function, whose maximum is located at the mean voting distance *ρ*_*m*_. Therefore, *ρ*_*m*_ can be obtained by fitting a quadratic function using the voting values in each column of the 2D accumulator.

In column *θ*_*i*_ of the 2D accumulator, all cells with nonzero votes are searched, and a quadratic function *f* is fitted to the data pairs (*H*^2^, *ρ*). The fitted function is denoted as

(3) $$\begin{array}{c} f:H^{2}\left(\rho ,\theta \right)=a_{2}\rho^{2}+a_{1}\rho +a_{0}. \end{array}$$

Figure 5 shows an example of the quadratic function fitting. The mean voting distance is determined by

(4) $$\begin{array}{c} \rho_{m}=\rho |\frac{\partial f}{\partial \rho }=0. \end{array}$$

### 2.4. Linear Function Fitting

For each voting angle *θ*, the computed mean voting distance *ρ*_*m*_(*θ*) is located at *ρ* whose voting value is the maximum. Following Figures 3 and 4, the line corresponding to maximum voting value passes through the center of the circular region, which means the center (*x*_0_, *y*_0_) of a cloud cluster always votes for the distance *ρ*_*m*_; therefore, there is the following formula:

(5) $$\begin{array}{c} \rho_{m}\left(\theta \right)=x_{0}\cdot \cos\;\theta +y_{0}\cdot \sin\;\theta . \end{array}$$

Thus, the relationship between the computed mean voting distance *ρ*_*m*_(*θ*) and the voting angle *θ* is a sine function, whose coefficients rely on the coordinates (*x*_0_, *y*_0_) of the region center. The center can be calculated by fitting a sine function. In order to calculate the center coordinates, conveniently, the sine function is linearized as

(6) $$\begin{array}{c} \frac{\rho_{m}\left(\theta \right)}{\cos\;\theta }=x_{0}+y_{0}\cdot \tan\;\theta . \end{array}$$

Thus, the functional relationship between *ρ*_*m*_(*θ*)/cos(*θ*) and tan(*θ*) is linear. We fit a linear function *g* using data pairs (*ρ*_*m*_(*θ*_*i*_)/cos(*θ*_*i*_), tan(*θ*_*i*_)). When the voting angles equal 40°, 48°, 56°, 64°, 72°, 80°, 88°, and 96°, the corresponding data pairs (*ρ*_*m*_(*θ*_*i*_)/cos(*θ*_*i*_), tan(*θ*_*i*_)) are shown in Table 1, and the linear function fitting is illustrated as Figure 6. In addition, to avoid the setting of *θ* to 90°, *θ* is often sampled at the discrete values around 90°.

The center coordinates (*x*_0_, *y*_0_) of the cloud cluster happen to be the fitted coefficients. The calculated center of the tropical cyclone is labeled in Figure 7.

## 3. Results

### 3.1. Implementation Details

The dataset used to test the proposed method is from Meteorological Satellite Observation Images of Typhoon Saomai (No. 200608) and Maria (No. 201808) provided by the Japan Meteorological Agency (JMA). Both the visible images and the infrared images are tested. With the satellite observation images, the cloud cluster of the tropical cyclone is extracted and its center is located.

The satellite cloud images are segmented using seed expanding techniques and threshold constraints. The segmented cloud cluster with the most pixels is recognized as the tropical cyclone; its center is calculated by voting and fitting. The center location results on two visible images and two infrared images are shown.

### 3.2. Experiments' Analysis

In Figure 8, it is noted that, despite of either the visible images or the infrared images, the proposed method is able to extract the regions of tropical cyclone. Based on the regions, the centers of the tropical cyclone can be further determined. In addition, the method can also deal with both eye cyclones and noneye cyclones. It is largely attributed to the fitting for the shape of the cyclone regions. Even though the shapes of tropical cyclones are irregular, the shapes are still approximated by circles. Once the circles are found, the centers can be determined. The located centers of typhoons are also compared with the Best Track (BT), and the averaged location errors are shown in Table 2. Because the size of typhoons is in itself large enough, these location errors can be tolerated. The experimental results show that the proposed center location method provides reliable estimates of tropical cyclone centers.

As illustrated in Figures 9 and 10, the segmentation of the typhoons region has great influence on the determination of the centers. When the segmented region covers most of the tropical cyclone, the shape of the cloud region is more likely to be a circle. As a result, the accuracy in the fitting of the circle is significantly improved. In Figure 7(a), while the tailor of the tropical cyclone is discarded, the segmentation maintains the central part of the tropical cyclone. The central part almost covers the whole tropical cyclone. Compared with the segmented cloud in Figure 9(a), the tropical cyclone in Figure 10(a) undergoes the deformation. It is obvious that the shape of the tropical cyclone in Figure 10(a) is irregular. It further causes the error in the estimation of the center of the tropical cyclone. Although it is inevitable for the error to be produced, the increase in the number of voting angle *θ* will reduce the error.

Like other methods for centers' location, the estimation of centers depends on the segmentation of the typhoons' region. The locating results are improved by using function techniques. A set of quadratic functions are fitted to voting values corresponding voting distances, and a linear function is fitted to mean voting distance with respect to the voting angle.

## 4. Discussion

In general, due to the existence of cloud tailors, small cloud clusters, and so on, it is difficult for the segmentation to generate the result of the tropical cyclone with the regular circular shape. Hence, it is important for the method to resist against the noises inherent to the segmentation results. The proposed method alleviates the errors in the estimation of centers caused by the irregular typhoons regions. Similar to other methods based on the morphological pattern analysis, the proposed method also relies on the organization structure of the tropical cyclone. Different with other methods, the proposed method uses not only skeleton points but also regional pixels. Therefore, the edge extraction, which is very sensitive to disturbance and noise, is not necessary. The proposed method is more robust than methods based on skeleton information. The robustness is largely attributed to the setting of multiple voting angles.

From Figures 11–18, the voting process of the parameters related to the circular region covering the typhoons region in Figure 2 is shown. At the same time, the fitting process is also given in these figures. In detail, a quadratic function is adopted to fit the relationship between the voting angle and the voting distance. To acquire the two-dimensional center location, it requires that at least two fitting functions are offered. In fact, the typhoons' region is often irregular, so the center location solved by two fitting functions is coarse. It means that more fitting functions are needed so as to give rise to an accurate estimation. In Figures 11–18, the voting angles are, respectively, sampled at 40°, 48°, 56°, 64°, 72°, 80°, 88°, and 96°. As a result, eight fitting functions are obtained. Among them, while the estimations of the voting distance in Figures 11 and 12 nearly distribute around the quadratic fitting functions, some points in Figures 13 and 14 significantly deviate from the fitting function. Along the lines with the angles 56° and 64°, the invagination of the shape inhibits the points from scattering around the quadratic functions. These points are more likely to be outliers. Hence, if only the points in Figures 13 and 14 are given, the quadratic functions estimated by these points cannot accurately represent the boundary enclosing the tropical cyclone. In Figures 17 and 18, *θ* is sampled at 88° and 96°, respectively, which are close to 90°. It avoids the setting of *θ* to the trivial value of 90°.

In the proposed method, the center location is usually located at the line with maximal voting distance. However, once the shape of the typhoon region is an irregular circle, it is possible for the estimated center to be far away from the real center of tropical cyclone. The usage of the fitting function removes the lines existing in the form of outliers. In Figure 13, the distribution of the points representing the voting distances in the proximity of the peak of the quadratic function is in chaos. Since that, in theory, the voting values corresponding to the regular circle should satisfy the quadratic function, the quadratic fitting to the function excludes those values that are not in favor of the estimation of the circle. Hence, it is obvious that the fitting to the quadratic function enhances the robustness of the estimation. The fitting functions with respect to more voting angles lead to more candidate centers. The regression over these centers can generate the reliable center. However, more fitting functions incur heavier computation burden, and it reduces the speed of finding the centers of tropical cyclones. Sometimes, the speed is important for the alert of the tropical cyclones.

In addition, the method is not sensitive to the type of images. Whatever the infrared image or the visible image is, the cloud cluster can be approximated as a near-circular region. Therefore, the center location method can be applied to the visible channel and infrared channel of meteorological satellite images.

## 5. Conclusions

An automatic method for cyclone center location is proposed based on regional pixels instead of skeleton points. The morphological structure of the tropical cyclone is modeled using the circular pattern. The skeleton extraction is avoided. By fitting a linear function, the center coordinates of the tropical cyclone happen to be the coefficients of the fitted function. The method can deal with both visible images and infrared images and both eye cyclones and noneye cyclones. The reliable estimates of tropical cyclone centers are obtained in spite of the variability of TC morphological structure in visible or infrared images. At present, the thresholds for the image binarization are manually selected. It cannot adapt itself to the segmentation requirement. In the future, it is possible for the adaptive image binarization to be brought into the image segmentation.

## Figures and Tables

**Figure 1:** The flowchart of the proposed algorithm.

**Figure 2:** Extraction of the cloud cluster.

**Figure 3:** Voting of regional pixels.

**Figure 4:** Voting value *H*(*θ*,*ρ*).

**Figure 5:** Quadratic function fitting.

**Figure 6:** Linear function fitting.

**Figure 7:** Center location.

**Figure 8:** Center estimates for eye and noneye cyclones in visible and infrared satellite images. (a) Satellite images in the infrared channel. (b) Satellite images in the visible channel.

**Figure 9:** (a) The region of the tropical cyclone is extracted from a visible satellite image by the segmentation. It is filled with the blue color. (b) The center of the tropical cyclone is determined based on the region of the tropical cyclone.

**Figure 10:** (a) The region of the tropical cyclone is extracted from a visible satellite image by the segmentation. It is filled with the blue color. (b) The center of the tropical cyclone is determined based on the region of the tropical cyclone.

**Figure 11:** The voting angle *θ* is set to 40°. When the voting distance *ρ* is 358.24, *H*(*θ*,*ρ*) reaches the peak.

**Figure 12:** The voting angle *θ* is set to 48°. When the voting distance *ρ* is 350.62, *H*(*θ*,*ρ*) reaches the peak.

**Figure 13:** The voting angle *θ* is set to 56°. When the voting distance *ρ* is 336.85, *H*(*θ*,*ρ*) reaches the peak.

**Figure 14:** The voting angle *θ* is set to 64°. When the voting distance *ρ* is 316.85, *H*(*θ*,*ρ*) reaches the peak.

**Figure 15:** The voting angle *θ* is set to 72°. When the voting distance *ρ* is 290.63, *H*(*θ*,*ρ*) reaches the peak.

**Figure 16:** The voting angle *θ* is set to 80°. When the voting distance *ρ* is 259.01, *H*(*θ*,*ρ*) reaches the peak.

**Figure 17:** The voting angle *θ* is set to 88°. When the voting distance *ρ* is 259.01, *H*(*θ*,*ρ*) reaches the peak.

**Figure 18:** The voting angle *θ* is set to 96°. When the voting distance *ρ* is 259.01, *H*(*θ*,*ρ*) reaches the peak.

**Table 1:** The relationship between *ρ*_*m*_(*θ*)/cos(*θ*) and tan(*θ*).

*θ*	40	48	56	64	72	80	88	96
*ρ*_*m*_	358.2352042	350.6212455	336.8496554	316.8497009	290.6307249	259.0087804	259.0087804	259.0087804
tan(*θ*)	0.839099631	1.110612515	1.482560969	2.050303842	3.077683537	5.67128182	28.63625328	−9.514364454
*ρ*_*m*_/cos(*θ*)	467.6428468	523.9952292	602.385426	722.7886763	940.5007823	1491.572119	7421.562053	−2477.878008

**Table 2:** The averaged errors of center location.

Tropical cyclones	Saomai (km)	Maria (km)
Averaged errors	18.62	20.56

## Data Availability

The raw/processed data required to reproduce these findings cannot be shared at this time as the data also form part of an ongoing study.
